The article "Potential Effects of Immunosuppression on Oxidative Stress and Atherosclerosis in Kidney Transplant Recipients" was published in 2021. Journal: Oxid Med Cell Longev.

# Potential Effects of Immunosuppression on Oxidative Stress and Atherosclerosis in Kidney Transplant Recipients

**DOI:** 10.1155/2021/6660846

**Published:** 2021-02-20

**Authors:** Marlena Kwiatkowska, Urszula Oldakowska-Jedynak, Ewa Wojtaszek, Tomasz Glogowski, Jolanta Malyszko

**Affiliations:** Department of Nephrology, Dialysis & Internal Diseases, The Medical University of Warsaw, Poland

## Abstract

Chronic kidney disease is a public health problem that, depending on the country, affects approximately 8–13% of the population, involving both males and females of all ages. Renal replacement therapy remains one of the most costly procedures. It is assumed that one of the factors influencing the course of chronic kidney disease might be oxidative stress. It is believed that the main mediators of oxidative stress are reactive oxygen species (ROS). Transiently increased concentrations of ROS play a significant role in maintaining an organism's homeostasis, as they are part of the redox-related signaling, and in the immune defense system, as they are produced in high amounts in inflammation. Systemic oxidative stress can significantly contribute to endothelial dysfunction along with exaggeration of atherosclerosis and development of cardiovascular disease, the leading cause of mortality in patients with kidney disease. Moreover, the progression of chronic kidney disease is strictly associated with the atherosclerotic process. Transplantation is the optimal method for renal replacement therapy. It improves better quality of life and prolongs survival compared with hemodialysis and peritoneal dialysis; however, even a successful transplantation does not correct the abnormalities found in chronic kidney disease. As transplantation reduces the concentration of uremic toxins, which are a factor of inflammation per se, both the procedure itself and the subsequent immunosuppressive treatment may be a factor that increases oxidative stress and hence vascular sclerosis and atherosclerotic cardiovascular disease. In the current work, we review the effect of several risk factors in kidney transplant recipients as well as immunosuppressive therapy on oxidative stress.

## 1. Introduction

Kidney transplantation (KTX) has evolved over the years to become the preferred means of renal replacement therapy for patients with end-stage renal disease, improving overall life expectancy and quality of life in these patients. Patient and graft survival rates are spectacular and usually provide excellent short-term and medium-term results. Despite this progress, there has been little improvement in the long-term renal graft and patient survival in a sense of various clinical complications that can develop due to the high complexity of this procedure [1–4]. It is well known that renal transplantation confers a survival advantage over dialysis treatment for patients with end-stage renal disease (ESRD) [1, 2]. However, the survival of transplant recipients is significantly lower than age-matched controls in the general population. The higher mortality in renal transplant recipients is, in part, due to comorbid medical illness, pretransplant dialysis treatment, and factors related to transplantation, including immunosuppression and other drug effects [3, 4]. Despite successful kidney transplantation, cardiovascular disease (CVD) remains the leading cause of morbidity and mortality in patients with chronic kidney disease (CKD) including predialysis, dialysis, and after renal transplantation subjects. Besides traditional risk factors, oxidative and nitrosative stress as well may contribute to the progress of CVD through the formation of atherosclerotic plaque [3, 4]. Oxidative stress, an imbalance between generation of oxidants and antioxidant defense system, is one of the major events which affects not only early posttransplantation phase but also graft and patient's long-term outcomes [5, 6]. This imbalance contributes to the elevated CVD morbidity and mortality as well as to the development of chronic allograft nephropathy, which is characterized by gradual decline in kidney function [7].

Kidney transplantation is aimed at restoring kidney function, but it incompletely mitigates pathological pathways and mechanisms of disease, such as chronic low-grade inflammation with persistent redox imbalance [8]. Among the other factors that can be involved in long-term kidney transplant complications as well as in elevated oxidative and nitrosative stress, immunosuppressive treatment has its role. After renal transplantation, there is an increase in oxidative phenomena related to endothelial dysfunction, inflammation, and atherosclerosis, which are responsible for both damage to the graft and cardiovascular complications, one of the major causes of patient death [9]. A number of studies demonstrate the prooxidant effects of both calcineurin inhibitors [9–11]; however, CsA has been described as a more potent oxidative stress inducer than TAC [12].

As we well know, the imbalance in the oxidant/antioxidant mechanisms leads to oxidative stress which plays a crucial role in vascular injury. The major mechanism leading to oxidative stress is the overproduction of ROS (reactive oxygen species). Disease entities such as hypertension and diabetes—the most common causes of ESRD—are characterized by high ROS production in the arterial walls [13, 14]. This underlies arterial remodeling and atherogenesis due to endothelial dysfunction and vascular inflammation. If we consider kidney failure as a consequence of these diseases, the farther kidney failure goes, the more pronounced the process becomes. Additional factors influencing the quality of the vessels will be the process of hemodialysis or aging in the pretransplant period itself. Detailed qualification of kidney transplant recipients and donors reduces the risk of failure, but there is no chance of organs deprived of this process. Surely, the transplant reduces the concentration of uremic toxins, which are a factor of inflammation per se, but both the procedure itself and the subsequent immunosuppressive treatment may be a factor that increases oxidative stress and hence vascular sclerosis and atherosclerotic cardiovascular disease (ASCVD).

## 2. Donor/Recipient Selection

### 2.1. Live > Death, Female > Male

A death donor kidney transplant is the most common organ donation procedure. Brain death, however, is associated with severe homodynamic disturbances [15], e.g., increasing blood pressure, decreasing cardiac output, and hormonal disturbances [16] which alter in tissue perfusion and activate the inflammatory process. The disturbances of hemodynamics and metabolism lead to ROS formation in the donor and correlate with ROS-mediated posttransplant kidney function. The significance of free radicals, measured by a quantitative evaluation of malondialdehyde (MDA), a stable product of lipid membrane peroxidation and total antioxidant status (TAS), was shown, i.e., by Kosieradzki et al. [17] in 2003. The gender of the recipients could be also important: some animal studies have shown an increased superoxide radical production and (in consequence) renal injury risk secondary to 17b-estradiol level, which may suggest greater oxidative stress in male recipients [18].

### 2.2. Less > More Risk Factors (including Age)

When performing a kidney transplant procedure in a patient with numerous risk factors, such as advanced pretransplant atherosclerosis, poorly controlled arterial hypertension, and especially advanced age of the recipient, it should be taken into account that vascular sclerosis could accelerate. The most commonly known age-associated changes in the endothelium are decreased activity (but not expression) of eNOS, increased arginase activity (decreased production and/or availability of NO), increased expression and activity of cyclooxygenases (COX) and their vasoconstrictors, and increased ROS production [19]. All this inevitably leads to an intensification of the existing oxidative stress and, consequently, to accelerated atherosclerosis, including vessel occlusion and graft ischemia; even if these changes were not significantly macroscopically expressed before transplantation [20], considering that atherosclerotic cardiovascular disease (ASCVD) is the leading cause of mortality [21], there is substantial risk of death-censored graft loss.

## 3. Transplant-Related Immune Activation

### 3.1. Role of CD8+ T Cell Activation

In human atherosclerosis lesions, we can find an increasing presence of CD8+ and CD4+ T cells. Some studies show that it may have an impact on the development of these lesions. Kyaw et al. [22] in their experiment proved that CD8+ T lymphocyte depletion has an intermediary influence on inflammatory cytokine TNF alpha and reduced atherosclerosis. Cochain et al. [23] drew a conclusion that CD8+ T cell promotes atherosclerosis because of controlling monopoiesis.

### 3.2. CMV Infection

Some factors during the posttransplant period, such as delayed graft function, cytomegalovirus infection, and microalbuminuria, which may damage renal function, produce a decreased antioxidant capacity (lower glutathione peroxidase (GPx)) [24]. Exposure of CMV before transplantation and posttransplant replication may have proatherogenic effects in relationship to the cellular immune response against CMV antigens. Ducloux et al. reported that CMV infection is associated with an accumulation of CD57+CD28-CD8+ T cells and divided patients into 3 groups: CMV negative, CMV positive without replication after Tx, and those with presented CMV replication after transplantation. The frequency of the presence of CD57+CD28-CD8+ T cells was highly related with the incidence of atherosclerotic events [25]. Interestingly, these terminally differentiated T cells are increased also in patients with ESRD (pretransplantation period) and IV stage CKD and they also correlate with CMV seropositivity. This might be the premature T cell aging effect, and it seems to be an unmodifiable factor even after successful kidney transplantation [25, 26].

### 3.3. Role of Allogenic Stimulation

In reference to the expected proatherogenic correlation between circulating CD57+CD28-CD8+ T cells and repeated stimulation of viral antibodies, there might be a relationship with HLA mismatch number and atherogenic-related events. In the cohort study analysis, Ducloux et al. observed higher risk in groups with increased points of HLA noncompliance. They assessed it as an independent risk factor of atherosclerosis [27]. As discussed above, atherosclerosis and cardiovascular diseases are associated with both the so-called traditional risk factors such as diabetes, hypertension, broadly understood endothelial dysfunction, and nontraditional risk factors such as oxidative stress (OS). We have increasing possibilities of biochemical, physical, and cellular evaluation of the impact of individual procedures, including immunosuppressive treatment, on the development of both oxidative stress itself and atherosclerosis—a consequence of OS and other components. In the case of oxidative stress, the most frequent biochemical factors assessed are TAC (total antioxidant capacity), MDA (malondialdehyde), GSH (glutathione), SOD (superoxide dismutase) activity, GPx (glutathione peroxidase) activity, CAT (catalase) activity, or oxLDL (oxidized LDL). SOD, GPx, and CAT are antioxidant enzymes; the concentration of which in patients with CKD is reduced and stage dependent. The improvement of glomerular filtration, a reduction in the concentration of uremic toxins, and other positive effects of KTX are followed by an increase in antioxidant factors; however, they do not reach the values observed in healthy individuals [28]. To evaluate atherosclerosis in patients after kidney transplantation, we can measure carotid intima media thickness (IMT) with ultrasound. There is a positive correlation between IMT and increased cardiovascular risk. An independent predictor of cardiovascular disease is also arterial stiffness—correlated with increased intravascular thrombosis due to some drug toxicity. This factor can be evaluated by measuring augmentation index and pulse wave velocity (PWV) [29].

### 3.4. Overview of Drugs Currently Used in Renal Transplantation

The current management of the renal transplant recipients using maintenance immunosuppression therapy is multimodal where most immunosuppressive regimens generally include a calcineurin inhibitor plus an adjunctive antiproliferative agent and steroids. The addition of induction therapy with a variety of monoclonal or polyclonal antibodies provides a more potent immunosuppression, and its use is more relevant in patients with a high immunological risk. More recently, mammalian target of rapamycin inhibitors has been incorporated in different protocols.

Immunosuppressive agents used in immunosuppressive therapy can be classified into three categories: induction therapy, maintenance therapy, and treatment for rejection.

Immunosuppressive medication can be divided into several subgroups; the most common are as follows:

(1) Drugs that inhibit the production of cytokines involved in the activation of cells and their clonal expansion.
  - Calcineurin inhibitors (CNI): cyclosporine A (CsA) and tacrolimus (TAC)
(2) Inhibitors of the proliferation signal
  - Mammalian target of rapamycin inhibitors (mTORi): sirolimus (SIR) and everolimus (EVERL)
(3) Drugs that inhibit cell division
  - Nonselective: azathioprine (AZA)
  - Selective: mycophenolate mofetil (MMF)
(4) Other drugs
  - Costimulant inhibitor: belatacept
  - Lymphodepletive therapy: ATG (antithymocyte globulin)
  - Anti-CD20 chimeric human and mouse monoclonal antibody: rituximab

## 4. Influence of Selected Groups of Drugs on Oxidative Stress and Atherosclerosis

### 4.1. Calcineurin Inhibitors (CsA, TAC)

Calcineurin inhibitors (CNIs) such as CsA and TAC are the main immunosuppressive drugs used to prevent the rejection in solid organ transplant recipients. Long-term treatment with CNIs increases the risk of adverse effects such as malignancy, chronic allograft dysfunction, and cardiovascular risk factors in this clinical population. In patients after transplantation treated with CNI, the most common complications are arterial hypertension secondary to endothelial damage and dysfunction causing vasoconstriction. They are also promoted intravascular fibrosis leading to increased arterial stiffness (chronic toxicity). In addition, there is evidence that CNI causes direct vascular toxicity by damaging vascular smooth muscle cells (VSMCs) [20–22]. Vascular damage leads to the decrease of renal function, which means CNIs have a potential nephrotoxicity effect [30, 31].

Also, they may lead to free radical overproduction [9–12]. Some authors confirmed that TAC patients have lower production of free radicals than patients on CsA-based regimen [32]. In spite of that, others conclude that there is no difference in oxidative stress parameters between the two immunosuppressive treatments [33].

Tacrolimus has a better cardiac-lipid profile than cyclosporine A. Some reports about the beneficial effect of tacrolimus on the level of oxidative stress in the organism have appeared. In particular, in vitro studies and animal tests indicate antioxidative properties for tacrolimus. Decreases in parameters of oxidative stress, such as the concentration of malondialdehyde (MDA), the activity of myeloperoxidase (MPO), and neutrophilic infiltration, have been observed after treatment. In in vitro studies on endotheliocytes, tacrolimus induced oxidative stress more weakly than other medications and was the only one that did not increase the production of nitric oxide (NO). The protective effect of tacrolimus on inflammatory response in rat liver during ischemia-reperfusion injury was also described. Findings in renal transplant recipients are not so clear and even indicate that the influence of tacrolimus on the activity of antioxidative enzymes in the kidneys may be involved in side effects of tacrolimus.

Moreno et al. studied 67 stable kidney transplant patients treated with calcineurin inhibitors who were not receiving cholesterol-lowering therapy and 14 healthy subjects. They demonstrated that the oxidative status did not differ between the cyclosporine and tacrolimus cohorts. Furthermore, transplanted patients showed a higher oxidative status (MDA increase and GPx decrease) than healthy subjects [24].

Recent studies have suggested that increased plasma malondialdehyde (MDA) levels are a consequence of specific immunosuppressive therapies. The study of Perrea et al. showed that immunosuppressive combined therapy with CyA was associated with the high values of MDA that were measured posttransplant. Moreover, this study provided strong evidence that tacrolimus is significantly associated with improved free radical metabolism [32].

### 4.2. Mechanisms

The research group Rodriguez-Diez et al. assessed the effects of CNI on murine endothelial cells. They observed dose-dependent upregulation of the synthesis nuclear factor kappa-light-chain enhancer of activated B cell- (NF-*κ*B-) dependent chemokines such as IL-6 and TNF-alpha. Moreover, both substances CsA and TAC induced the synthesis of important vascular proinflammatory cytokines IL-6 and TNF-alpha which in turn cause inflammation and endothelial damage [34].

The impact of NFK on heart disease has been shown, among others, in Van der Heiden et al.'s study [35].

The key events mediating between CNI and inflammation on endothelial cells are Toll-like receptor signaling (TLRs). The vascular response to injury develops through signaling mediated by TLRs and is a key component of innate immunity.

To assess the effect of TLRs on NF-*κ*B, the effects of CNI in mice with the MyD88 adapter protein gene silenced were studied, which prevented the synthesis of agonists in the TLR activation pathway. Administration of TAC to such a modified organism resulted in the much lower activity of the NF-*κ*B-dependent pathway.

As TLR4 is particularly important in the development of vascular diseases, in the next step, pharmacological signal transmission, specifically from the intracellular part of TLR4, was blocked pharmacologically. After analysis, a decreased expression of genes leading to the synthesis of proinflammatory cytokines was found [34].

In addition, decreased ROS production was also noted in VSCM cells and endothelial cells, which means reducing the oxidative stress and its consequences described in the previous paragraphs.

Data on whether any of the CNIs have a lower proinflammatory effect are inconclusive; in some, there are data that CsA increases the risk of OS [36]; in others, the impact of both CsA and TAC on OS is assessed as similar [28, 37].

### 4.3. CNI (CsA) vs. Belatacept

Due to the CNI side effects, including nephrotoxicity, some analyses are trying to bring new, alternative solutions to immunosuppression—with a lower intensity of vascular (and as a consequence renal) side effects. Costimulation inhibitor belatacept (BELA), one of the promising ones, although not yet registered in all countries (e.g., not available in Poland), is registered in Europe and the USA in 2011 (Nulojix BMS). Pooled analysis of the BENEFIT study and BENEFIT-EXT showed, among others, belatacept (costimulant inhibitor) as an alternative which is associated with less hypertension, hyperlipidemia, and NODAT (new-onset diabetes) [37–41]. In a 46-patient study organized by Seibert et al. [38], PWV was assessed in two groups, with a similar profile of comorbidities—23 participants treated with CsA and 23 with belatacept. In the measurement of brachial blood pressure, serum lipid level was also used for the assessment. Statistically, significantly higher systolic blood pressure and faster heart rate were observed in the group treated with CsA, as is the rate of NODAT and level of serum lipids. PWV and augmentation pressure were lower in patients receiving belatacept, but this did not show a statistically significant difference.

The authors believe that the lack of unequivocal benefit associated with the use of belatacept, despite its lower vasoconstriction potential, thus a lower incidence of HT and other complications, may be associated with a too small control group and too short observation time. Therefore, it seems justified to extend the study to new participants with an extension of the study duration. Looking at the limited data, it seems that it has the potential to reduce atherosclerosis and the incidence and death of cardiovascular diseases.

### 4.4. Mammalian Target of Rapamycin (mTOR)

mTOR is a subunit of 2 distinct multicomplexes (mTORC1 and mTORC2), which play a crucial role in various processes, e.g., cell proliferation, protein synthesis, and glycolysis. Activation of mTORC1 is triggered by several stimuli, such as availability of nutrients and ATP, growth factors, and oxidative stress [42]. Systemic lupus erythematosus (SLE) patients exhibit various disturbances in the immune system that can be linked to, among other things, mitochondrial dysfunction of T cells, which results in increased generation of ROS and glutathione (GSH) depletion. Subsequent oxidative stress-related mTORC1 activation leads to dysregulation of various T cell subpopulations [43]. Interestingly, according to a study conducted by Lai et al., treatment with NAC increases levels of GSH and reduces mTOR activation in peripheral blood lymphocytes, which leads to improvement in disease activity scores in SLE patients [44]. In kidney transplant recipients, ischemia-reperfusion injury (IRI) is a vital problem that is responsible for delayed graft function as well as immune activation, which in turn results in acute rejection and chronic graft nephropathy. Initial consequence of IRI is associated with oxygen depletion and production of ROS in mitochondria of kidney tubular cells. The resulting oxidative stress has a damaging effect on kidney tissue and creates a proinflammatory environment, which even after restoration of sufficient blood flow continues to exert detrimental influence, promoting apoptosis, inflammation, and fibrosis [45]. Therapeutic strategies of targeting mTOR in order to ameliorate IRI have been evaluated in various animal models. Kezić et al. evaluated the effect of everolimus on IRI-associated NF-kappa B activity, production of IL-1-beta, TNF-alpha, and IL-10. It turned out that everolimus-treated animals displayed higher concentration of proinflammatory cytokines in the early phase of IRI [46]. An earlier study conducted by Suyani et al. compared, among other things, the effect of everolimus on levels of malondialdehyde (MDA), superoxide dismutase (SOD), and myeloperoxidase (MPO) in rats subjected to IRI. While levels of MDA and MPO were significantly lower in the everolimus group compared with the nontreated group, which indicated lower lipid peroxidation and decreased neutrophil and mononuclear infiltration, SOD activity remained low in both groups, corresponding with SOD depletion associated with oxidative stress [47]. The results proved to be inconclusive—on the one hand, mTOR inhibition immediately after transplantation may interfere with recovery of graft function likely as a result of antiproliferative and proapoptotic effect of mTORi, as well as overactivation of autophagy, while on the other hand long-term beneficial effect of mTORi on oxidative stress and immune activation improved outcomes during the recovery phase [48, 49].

The currently available studies assessing the impact of mTORis on cardiovascular diseases do not provide conclusive data. This drug group is associated with an increased risk of hyperlipidemia, endothelial dysfunction, and diabetes, which are known risk factors for both atherosclerosis and heart disease [50, 51]. On the other hand, part of the research on animals suggests the antiatherosclerotic effects of mTOR [52]. Taking into account these discrepancies in the data, e.g., in a small study by the team of Szymczak et al. [53], the effect of using sirolimus and tacrolimus versus CNI/MMF was assessed in a group of 44 patients after KT. Analysis included laboratory data such as serum lipid level (LDL, HDL, and TG), uric acid, and glycated hemoglobin. The severity of atherosclerosis was assessed by ultrasound IMT measurement—wall thickening > 14 mm over a length > 10 mm was treated as an atherosclerotic plaque. The results of this study revealed higher levels of total cholesterol and triglycerides in patients taking mTOR (statistically significant difference) compared to those on CNI. Both groups received statins. There were statistically more cases of NODAT in the mTORi group (34% vs. 25%). This translated into an increased risk of myocardial infarction per patient per 5 years. However, no significant difference was found in the mean IMT thickness [53]. Therefore, this was the opposite conclusion compared to the studies proving the prevention of coronary artery disease in patients after heart transplantation receiving mTOR, including antirestenotic activity of the stent achieved in the coronary arteries [54, 55]. It seems impossible to extrapolate these achievements in terms of the group of patients after KTX. The reasons for this include a greater decrease of glomerular filtration, disturbances in calcium-phosphate balance, and a more frequent tendency to hypertension occurring in kidney transplantation recipients.

Steroids and calcineurin inhibitors inhibit inducible nitric oxide, thus helping to determine endothelial dysfunction associated with onset and progression of atherosclerosis and vascular calcification. Much more complex are the vascular effects of mTOR inhibitors. Rapamycin inhibits smooth muscle cell proliferation, while everolimus impairs the vasoactive and antithrombotic function of endothelial cells [56]. Some studies suggest a relationship between vascular calcification and impaired bone metabolism as well as an involvement of immunosuppressive drugs on expression, regulation, and function of RANKL, RANK, and osteoprotegerin (OPG) system working in the skeletal and vascular systems. In particular, sirolimus inhibits osteoclast formation, unlike steroids and cyclosporine [57].

mTORis, in their pathomechanism of action, inhibit the formation of atherosclerotic plaques—i.e., they inhibit macrophages and VSMC proliferation, but this is a beneficial effect of vessels with plaque forming, not existing ones. Despite reports on the beneficial effect of sirolimus in aortic stiffness [58] by reducing oxidative stress and plasma endothelin-1 concentration, the advantage over CNI in terms of atherosclerotic complications cannot be unequivocally recognized—similar to other groups of drugs, patients treated with mTOR have an increased cardiovascular risk and require intensive monitoring.

### 4.5. Lymphodepletive Therapy: ATG Treatment

Antithymocyte globulin (ATG) for many years was used as an immunosuppressive treatment in solid organ transplantation. These polyclonal antibodies lead to T cell depletion and induce wide and persistent changes in T cell subpopulations including CD8+ T cell expansion [25].

As previously described, the repopulation of T cells with a predominance of CD8+ T cells is clinically correlated with an increased risk of atherogenesis. Considering the additional effect of CMV infection in transplant patients, Havenith et al. [59] in their work noted a significant acceleration of atherosclerosis in CMV-positive patients taking ATG, with no significant difference in CMV I patients. Therefore, ATG should be taken into account in the mechanism of atherosclerotic lesion formation as a cofactor in combination with CMV infection, without a significant effect in patients without this burden.

### 4.6. Rituximab

Rituximab is a chimeric human and mouse monoclonal antibody that reacts with CD20 antigen presented on pre-B and mature B lymphocytes. Therefore, it is often used in transplantation for pretransplant desensitization in patients with HLA or ABO incompatibility and posttransplant treatment of acute antibody-related rejection or lymphoproliferative diseases, including posttransplant [60]. Thus far, the effect of rituximab on the formation of atherosclerotic plaques in patients with rheumatic diseases has been reported. There are also studies, mainly with small groups of subjects, assessing the same effect in transplant patients. They are based on the qualitative and quantitative evaluation of biomarkers related to the atherosclerosis process—e.g., a study by Aliyeva et al. [61] assessed the presence and abundance of factors such as Il-10, TNF-alpha, and CD56+ NK (natural killer) cells. What draws attention are two conflicting effects on vascular sclerosis. As in the case of ATG, there is a significant correlation with CMV infection—here, however, rituximab is not so much a cofactor as it increases the risk of CMV infection/reinfection and related vascular complications. At the same time, there are (limited) data that the use of rituximab has a positive effect on the concentration of IL-10 and anti-oxLDL, which reduces systemic inflammation. However, these are data for patients with rheumatoid arthritis. These data do not currently support patients receiving rituximab for kidney transplantation (higher baseline cardiovascular risk?). Due to the existing antiatherogenic potential, a positive effect of CMV prophylaxis combined with rituximab is possible, but it requires a further randomized and larger group of patient trials [61].

## 5. Final Considerations and Future Perspectives

Kidney transplantation is the treatment of choice for end-stage renal disease. Despite the fact that successful kidney transplant improves the quality of life and reduces mortality for most patients relative to those on maintenance dialysis, immunosuppressive therapy bears the risk of infection, malignancy, and cardiovascular disease. Immunosuppression maybe also a factor that increases oxidative stress and hence vascular sclerosis and atherosclerotic cardiovascular disease.  Table 1 presents an overview of published data of the studies designed to assess the oxidative state of renal transplant patients. Oxidative stress, an imbalance between the generation of oxidants and antioxidant defense system, is one of the major events which affects not only early posttransplantation phase but also graft and patient's long-term outcomes. This imbalance contributes to the elevated cardiovascular morbidity and mortality as well as to the development of chronic allograft nephropathy, which is characterized by gradual decline in kidney function leading finally to graft loss. There is no ideal immunosuppressive regimen for kidney transplant recipients; all schemes have unwanted side effects. However, it is a price to pay to have a better and longer life. Reactive oxygen species can be removed by our intrinsic enzymatic system. In addition, a range of antioxidant chemical agents can be introduced to the organism, e.g., in a diet. Antioxidant therapies have not become a standard of care in renal patients up to date and more investigations are needed. It mainly remains unknown how antioxidant treatment can potentially alter the progression of chronic kidney disease itself. We also have to take into consideration not only kidney function but also the effects of immunosuppression on the biomarkers of oxidative stress. In clinical research, antioxidant therapies require more time to confirm the applicability of various antioxidant agents as effective treatment methods, in particular in heterogeneous vulnerable populations. The most important question of correlation between disturbance in the balance of pro- and antioxidant systems and its influence on the development and progression of chronic kidney disease still remains unanswered, so an era of tailored immunosuppressive therapy for kidney transplant recipients. Personalized medicine in the field of clinical transplantation is eagerly awaited; however, due to pandemic, it may be postponed due to many reasons (shortage of donors, shortage of financial resources, other priorities such as vaccines, new antiviral drugs, etc.).

## Figures and Tables

**Table 1:** Overview of published data of the studies designed to assess the oxidative state of renal transplant patients.

Study	Objective	Results/conclusions
Moreno et al. [24]	The study was designed to assess the oxidative state of transplant patients with stable renal function; 67 stable kidney transplant patients treated with calcineurin inhibitors were studied.	Transplanted patients showed a higher oxidative status (MDA increase and GPx decrease) than healthy subjects. The oxidative status did not differ between the cyclosporine and tacrolimus cohorts.

Ruiz et al. [6]	The study was designed to determine the relationship between the presence of carotid artery lesions and oxidative parameters in 50 renal transplanted patients with stable renal function.	The serum GPx level among patients without atheroma plaques, calcification, or stenosis was higher than in those with ultrasound signs.

Perrea et al. [32]	The study included 26 renal transplant patients, treated with a different combination of immunosuppressive agents: CyA-MMF-PRED-basiliximab and TAC-MMF-PRED-daclizumab. Plasma MDA levels were measured before transplantation and 1 and 6 months after TX.	Levels of MDA were increased before the transplantation in all renal patients. Immunosuppressive combined therapy with CyA was associated with the high values of MDA posttransplant. This study provides strong evidence that TAC is significantly associated with improved free radical metabolism.

Zadrazil et al. [33]	AOPP and TAS were evaluated in transplanted patients on different calcineurin inhibitors. 35 patients were treated with CsA and 33 with TAC.	No significant differences in AOPP and TAS were found with respect to treatment. The only exception was the higher mean concentration of AOPP at month 1 in recipients treated with CsA.

Szymczak et al. [53]	The aim of this study was to compare the effect of immunosuppressive regimens using either mTORi or CNI on the risk of atherosclerosis in RARs. The study involved 24 RARs treated with mTORi and 20 RARs treated with immunosuppressive regimen based on CNI. Carotid atherosclerosis was evaluated by measurement IMT of the common and internal carotid artery walls and detection of carotid plaques by high-resolution ultrasonography. The study was performed 3-24 years after TX.	The mTORi group showed higher level of TC, LDL-C, and TG. Posttransplant diabetes developed in 34% of the mTORi group compared with 25% in the CNI group. There was no beneficial effect of immunosuppressive treatment with mTORi on carotid atherosclerosis in RARs.

Joannidès et al. [58]	The study was designed to evaluate whether or not CsA-free immunosuppressive regimen based on SRL prevents aortic stiffening and improves central hemodynamics in RARs. 44 patients enrolled in the trial were randomized at week 12 to continue CsA or switch to SRL, both associated with MMF. cSBP, cPP, AIx, and PWV: aortic stiffness was blindly assessed at W12, W26, and W52 together with ET-1, TBARS, and SOD and CT erythrocyte activities.	At W12, there was no difference between groups. At follow-up, PWV, cSBP, cPP, and AIx were lower in the SRL group. In parallel, ET-1 decreased in the SRL group, while TBARS, SOD, and CT erythrocyte activities increased in both groups but to a lesser extent in the SRL group. These results demonstrate that a CsA-free regimen based on SRL reduces aortic stiffness, ET-1, and oxidative stress in RARs suggesting a protective effect on the arterial wall that may be translated into cardiovascular risk reduction.

Juskowa et al. [5]	The study was designed to examine markers of lipid peroxidation and antioxidant potential in the blood (serum, plasma, and RBC) of 51 RARs and sex-matched volunteers as a control group (C). RARs were divided into two subgroups: RARs-A (*n* = 28) were treated with triple-drug therapy including CsA and RARs-Z (*n* = 23) were on double-drug regimen: PRED and AZA. We used several automated assays to estimate MDA, TRAP, GPx, GSH, SOD, CAT, vit. E, and lipid profiles.	Patients of RARs-A were found to have significantly elevated triglycerides, cholesterol-LDL, MDA, and TRAP and decreased activity of RBC glutathione peroxidase as compared with those of RARs-Z and group C. In conclusion, our data show that oxidative stress (with prooxidant effect of CsA partly at least), with reduced antioxidant potential of defense system, is associated with KTX.

Chrzanowska et al. [10]	The aim of the study was to analyze the relation between total antioxidant capacity and immunosuppressive therapies, renal function, and hematocrit in kidney transplant patients. The study included 46 adult patients following renal transplantation, treated with different combinations of immunosuppressive agents: with CsA (*n* = 23) or TAC (*n* = 15).	There was a significantly negative correlation between TAOC and plasma creatinine and a positive correlation between TAOC and creatinine clearance or hematocrit in patients treated with TAC but not with CsA. Immunosuppressive therapy with CsA was associated with higher TAOC. Anemia can be an independent risk factor for an increase of oxidative stress. TAOC was positively associated with renal function in patients treated with TAC.

Vural et al. [11]	23 KTX patients were included in the study. MDA, plasma selenium (se), GSH-Px, SOD, EZn, and ECu levels were studied before and in the 1st, 3rd, 7th, 14th, and 28th days after TX. 11 recipients were treated with CsA whereas 12 patients were treated with TAC.	The GSH-Px, SOD, ECu, EZn, and selenium levels were lower and MDA levels were higher in patients than controls before TX. MDA levels decreased and SOD, GSH-Px, ECu, and EZn levels increased in parallel to the decrement of serum creatinine levels following KTX. No difference was found among the patients regarding the treatment regime. The study data suggest that the improvement in oxidative state parameters begins at the first day of KTX and continues at the 28th posttransplant day in living donor TX.

Cofan et al. [12]	The objective of this study was to analyze the effect of converting from cyclosporine to tacrolimus on lipoprotein oxidation in renal transplant recipients. 12 recipients were studied treated with a CsA-MMF-PRED combination that was converted to TAC-MMF-PRED.	The conversion to TAC resulted in significant decrease in TC levels and produced a nonsignificant decrease in Ab-oxLDL. In renal TX, TAC therapy was associated with a better lipid profile and lower in vivo LDL oxidation when compared with CsA treatment.

Ab-oxLDL: oxidized LDL autoantibodies; AOPP: advanced oxidation protein products; AIx: augmentation index; AZA: azathioprine; CAT: catalase; CNI: calcineurin inhibitor; Cr: creatinine; CsA: cyclosporine A; ECu: erythrocyte Cu; ET-1: endothelin-1; EZn: erythrocyte Zn; GPx: glutathione peroxidase; GR: glutathione reductase; GSH: glutathione; GSH-Px: erythrocyte glutathione peroxidase; IMT: intimal media thickness; KTX: kidney transplant patients; LDL: low-density lipoprotein cholesterol; MDA: malondialdehyde; mTORi: mammalian target of rapamycin inhibitors; MMF: mycophenolate mofetil; OS: oxidative stress; PRED: prednisone; SOD: superoxide dismutase; cPP: pulse pressure; PWV: aortic stiffness carotid-to-femoral pulse-wave velocity; RARs: renal allograft recipients; cSBP: carotid systolic blood pressure; SIR: sirolimus; TAC: tacrolimus; TAOC: total antioxidant capacity; TAS: total antioxidant status; TC: total cholesterol; TG: triglycerides; TBARS: thiobarbituric acid-reactive substances; TRAP: total radical-trapping antioxidant potential; TX: transplantation.
